The article "Differential Diagnosis of Hemophagocytic Syndrome by 18F-FDG PET/CT: A Meta-Analysis" was retracted in 2023. Reasons: signs of a paper mill; suspected computer-generated content; unreliable results or conclusions; lack of ethics approval or compliance.

# Differential Diagnosis of Hemophagocytic Syndrome by ^18^F-FDG PET/CT: A Meta-Analysis

**DOI:** 10.1155/2022/4448993

**Published:** 2022-01-29

**Authors:** Jun Zhang, Bang He, Jian Wang, Caiyun Ying, Lingfeng Zeng, Shiyi Zheng

**Affiliations:** ^1^Department of Neurology, Chengdu Xindu District People's Hospital, Chengdu, Sichuan, China; ^2^Department of Nuclear Medicine Sir Run Run Shaw Hospital School of Medicine, Zhejiang University, Hangzhou, Zhejiang, China; ^3^Department of Radiology, The First People's Hospital of Chongqing Liang Jiang New Area, Chongqing, China; ^4^Department of Medicine, The Second Xiangya Hospital, Central South University, Changsha, Hunan, China

## Abstract

Hemophagocytic syndrome (HPS) is a rare disease in clinical practice, and there are often cases of delayed diagnosis. At present, researchers have applied ^18^F-FDG PET/CT in the differential diagnosis of HPS, but no consensus has been formed. Therefore, this study aims to systematically evaluate the application value of ^18^F-FDG PET/CT in the diagnosis of HPS patients. PubMed, Embase, Cochrane Library, Chinese National Knowledge Infrastructure (CNKI), Wangfang database (Wangfang), and Chinese Biomedical Network (CBM) were searched to collect the relevant studies of ^18^F-FDG PET/CT in the diagnosis of HPS. Data from the articles were screened and extracted for meta-analysis using Stata16.0 software. A total of 10 retrospective studies, including 300 patients, were included in this meta-analysis. The meta-analysis results showed that the pooled sensitivity was 0.82 (95% CI: 0.67–0.95), specificity was 0.72 (95% CI: 0.51–0.86), positive likelihood ratio was 2.89 (95% CI: 1.46–5.75), positive likelihood ratio was 0.25 (95% CI: 0.12–0.54), diagnostic odds ratio was 2.89 (95% CI: 1.46–5.75), and AUC was 0.84 (95% CI: 0.81–0.87). The SUVmax in the liver, spleen, lymph nodes, and bone marrow of HPS patients was greater than 2.5, and the SUVmax in the spleen, lymph nodes, and bone marrow of malignant HPS patients was higher than that of benign HPS patients. The difference was statistically significant (*P* < 0.05). According to the existing literature evidence, ^18^F-FDG PET/CT is an effective method for diagnosing HPS.

## 1. Introduction

Hemophagocytic syndrome (HPS), also known as hemophagocytic lymph hyperplasia, is a clinical illness in which excessive inflammatory responses are induced by primary or secondary immune system disorders (HLH). HPS can occur at any age, but most cases occur in adults [1]. HPS is a rare disease, and studies have reported that the annual incidence of HPS is about 1 in 800,000, with a male to female ratio of about 1 : 7. Still, due to the secretion of large amounts of inflammatory factors, it can also threaten the patient's life in severe cases, with a mortality rate as high as 40% [2, 3]. The main clinical manifestations in patients with HPS are intermittent fever, hepatosplenomegaly, lymphadenopathy, and pancytopenia [4, 5]. However, the clinical manifestations of HPS are diverse and lack specificity and usually mimic or overlap with the clinical manifestations of diseases such as systemic inflammatory response syndrome, multiple organ failure, and sepsis [6].

The article "Differential Diagnosis of Hemophagocytic Syndrome by 18F-FDG PET/CT: A Meta-Analysis" was retracted in 2023. Reasons: signs of a paper mill; suspected computer-generated content; unreliable results or conclusions; lack of ethics approval or compliance.

HPS mainly includes two types: primary and secondary. Primary HPS is caused by hereditary immune dysfunction, is known as familial hemophagocytic lymphohistiocytosis, and primarily occurs in infants [7]. Secondary HPS is mainly caused by malignant tumors, autoimmune diseases, and chronic viral infections and is less likely to be secondary to conditions such as chronic diseases (chronic nephritis, liver disease, diabetes, and chronic granulomatous diseases) and pernicious anemia [8–10]. Among the causes of secondary HPS, malignant tumors are the most common (about 45%), and most of them are hematological malignancies such as lymphoma, which occur less frequently in solid tumors [4], followed by infections, with Epstein-Barr virus infection being the most common [11]. Autoimmune disease-associated HPS is often associated with Kawasaki disease and systemic juvenile idiopathic arthritis in children and systemic lupus erythematosus, adult Still's a disease, and rheumatoid arthritis in adults [12]. Among the many causes mentioned above, HPS caused by hematologic tumors is the most common, and patients often have a worse prognosis. Therefore, early identification of tumor-associated HPS, timely intervention and avoidance of misdiagnosis, and delayed treatment are essential to improve the prognosis of patients. At present, many studies have explored the diagnosis of HPS. As a whole-body metabolic imaging, 18-fluorodeoxyglucose positron emission tomography/computed tomography (^18^F-FDG PET/CT) has recently been widely used in the diagnosis, staging, and efficacy evaluation of tumors, especially lymphomas, and in the diagnosis and treatment of fever of unknown origin and autoimmune diseases [13–16]. Whether the ^18^F-FDG PET/CT could be used for the diagnosis of hemophagocytic syndrome was under debate. The conclusion in previous studies was controversial, and the sample size was small. The meta-analysis could pool the studies of small sample size, and we could draw a stable conclusion by means of meta-analysis. This is the first meta-analysis to study the diagnosis of hemophagocytic syndrome by the ^18^F-FDG PET/CT [9, 17–25]. The ten studies included in this meta-analysis [26–28] were all relevant reports on the use of ^18^F-FDG PET/CT for the differential or diagnosis of HPS. The conclusions of the above 10 studies were conflict; therefore, the objective of the study was to evaluate the diagnostic performance of 18F-FDG PET/CT for the hemophagocytic syndrome.

The article "Differential Diagnosis of Hemophagocytic Syndrome by 18F-FDG PET/CT: A Meta-Analysis" was retracted in 2023. Reasons: signs of a paper mill; suspected computer-generated content; unreliable results or conclusions; lack of ethics approval or compliance.

## 2. Materials and Methods

### 2.1. Literature Search

PubMed, Embase, Cochrane Library, CNKI, Wangfang, and CBM were searched for relevant studies on 18F-FDG PET/CT for the diagnosis of HPS from database establishment to June 15, 2021, and the search languages were only Chinese and English. Search terms were “PET,” “PET/CT,” “PET-CT,” “Positron Emission Tomography-Computed Tomography,” “Hemophagocytic Lymphohistiocytoses,” “Hemophagocytic Lymphohistiocytosis,” “Hemophagocytic Syndrome,” “Infection-Associated Hemophagocytic Syndrome,” “Familial Hemophagocytic Lymphocytosis,” “Familial Hemophagocytic Lymphocytoses,” “Primary Hemophagocytic Lymphohistiocytosis,” “Primary Hemophagocytic Lymphohistiocytoses,” “Familial Erythrophagocytic Lymphohistiocytosis,” “Familial Erythrophagocytic Lymphohistiocytoses,” “Familial Histiocytic Reticulosis,” “Familial Histiocytic Reticuloses,” “Primary Hemophagocytic Hymphohistiocytosis,” “Primary Hemophagocytic Hymphohistiocytoses,” “Primary Hemophagocytic Hymphohistiocytoses,” “Familial Hemophagocytic Reticuloses,” “Familial Hemophagocytic Lymphohistiocytosis,” “Familial Hemophagocytic Histiocytosis,” “Familial Hemophagocytic Histiocytoses,” and “Familial Hemophagocytic Lymphohistiocytoses”. The retrieval formula is ((“Lymphohistiocytosis, Hemophagocytic”[Mesh]) OR ((((((((((((((((((((Hemophagocytic Lymphohistiocytoses[Title/Abstract]) OR (Hemophagocytic Lymphohistiocytosis[Title/Abstract])) OR (Hemophagocytic Syndrome[Title/Abstract])) OR (Infection-Associated Hemophagocytic Syndrome[Title/Abstract])) OR (Familial Hemophagocytic Lymphocytosis[Title/Abstract])) OR (Familial Hemophagocytic Lymphocytoses[Title/Abstract])) OR (Primary Hemophagocytic Lymphohistiocytosis[Title/Abstract])) OR (Primary Hemophagocytic Lymphohistiocytoses[Title/Abstract])) OR (Familial Erythrophagocytic Lymphohistiocytosis[Title/Abstract])) OR (Familial Erythrophagocytic Lymphohistiocytoses[Title/Abstract])) OR (Familial Histiocytic Reticulosis[Title/Abstract])) OR (Familial Histiocytic Reticuloses[Title/Abstract])) OR (Primary Hemophagocytic Hymphohistiocytosis[Title/Abstract])) OR (Primary Hemophagocytic Hymphohistiocytoses[Title/Abstract])) OR (Familial Hemophagocytic Reticuloses[Title/Abstract])) OR (Familial Hemophagocytic Lymphohistiocytosis[Title/Abstract])) OR (Familial Hemophagocytic Histiocytosis[Title/Abstract])) OR (Familial Hemophagocytic Histiocytoses[Title/Abstract])) OR (Familial Hemophagocytic Reticulosis[Title/Abstract])) OR (Familial Hemophagocytic Lymphohistiocytoses[Title/Abstract]))) AND ((“Positron Emission Tomography Computed Tomography”[Mesh]) OR ((((((PET-CT[Title/Abstract]) OR (PET-CT[Title/Abstract])) OR (Positron Emission Tomography-Computed Tomography[Title/Abstract])) OR (PET-CT[Title/Abstract])) OR (PET/CT[Title/Abstract])) OR (PET[Title/Abstract]))).

The article "Differential Diagnosis of Hemophagocytic Syndrome by 18F-FDG PET/CT: A Meta-Analysis" was retracted in 2023. Reasons: signs of a paper mill; suspected computer-generated content; unreliable results or conclusions; lack of ethics approval or compliance.

### 2.2. Inclusion and Exclusion Criteria

Inclusion criteria were as follows: (1) The types of studies selected for this meta-analysis were retrospective studies. (2) The experimental group of the study was patients with malignant HPS; the control group was patients with benign HPS. (3) The included studies needed to contain at least one of the following indicators: maximum standardized uptake value (SUVmax) of the liver, spleen, lymph nodes, and bone marrow and diagnostic efficacy of benign and malignant HPS. (4) The included study subjects were patients with a definite diagnosis of HPS, and the diagnostic criteria for HPS (5) The reported data in the literature are complete.

Exclusion criteria were as follows: (1) The results are not wholly statistically analyzed, or the relevant data are insufficient. (2) Published literature is repeated. (3) The study subjects are not HPS patients. (4) Studies are conference, meta-analysis, and review literature.

### 2.3. Literature Screening and Data Extraction

The retrieved literature was initially screened by two investigators independently according to the inclusion and exclusion criteria and then cross-checked. The controversial literature was evaluated by the third party and then unified by discussion. Two investigators extracted the relevant information of the included literature, including the first author, publication year, publication country, sample size, maximum standardized uptake value (SUVmax) of liver, spleen, lymph nodes, and bone marrow, and diagnostic efficacy of benign and malignant HPS.

### 2.4. Literature Quality Evaluation

Two investigators evaluated the quality of the included studies according to the quality assessment of diagnostic accuracy studies (QUADAS): the selection of patients, index tests, reference standards, processes, and time in the included studies were judged, and the judgment results included “yes,” “no,” and “unclear.” If all were “yes,” it was graded as grade A. If at least one was “unclear” and did not contain “no,” it was graded as grade B, and if any item was “no,” it was graded as grade C.

### 2.5. Statistical Methods

Meta-analysis was performed on the data using Stata16.0 software, weighted mean difference (WMD) was used for measurement data, and 95% confidence interval (CI) was used for interval estimation. The interval is computed at a designated confidence level. A 95% confidence level is most common, but other levels, such as 90% or 99%, are sometimes used. In this study, we have used the 95% confidence level to study and evaluate the application value of 18F-FDG PET/CT in the diagnosis of HPS. Between-study heterogeneity was determined by the *χ*2 test combined with quantitative analysis of *I*^2^. If *P* > 0.1 and *I*^2^ < 50%, it was considered that between-study heterogeneity was acceptable, and the fixed-effect model was used for meta-analysis; if *P* < 0.1 and *I*^2^ > 50%, it was deemed that between-study heterogeneity was significant, and random-effect model was used for analysis. The pooled sensitivity, specificity, likelihood ratio, and diagnostic odds ratio of the included studies were calculated. A summary receiver operating characteristic (ROC) curve fitting analysis was also performed to obtain Area Under Curve (AUC). The diagnostic efficacy was judged according to the AUC value, with AUC < 0.50 as too low diagnostic efficacy without clinical application value, 0.50 to 0.70 as low diagnostic efficacy, 0.71 to 0.90 as moderate diagnostic efficacy, and >0.90 as high diagnostic efficacy. Deek's linear regression analysis was used to evaluate publication bias, and *P* < 0.01 indicated the presence of publication bias.

The article "Differential Diagnosis of Hemophagocytic Syndrome by 18F-FDG PET/CT: A Meta-Analysis" was retracted in 2023. Reasons: signs of a paper mill; suspected computer-generated content; unreliable results or conclusions; lack of ethics approval or compliance.

## 3. Results

### 3.1. Literature Search and Screening Results

In this meta-analysis, 321 relevant pieces of literature were obtained through preliminary retrieval, 207 were left after excluding repeated literature, 42 were left after excluding irrelevant study through a reading title, and ten were left after excluding literature including abstract, animal study, and review through reading the full text. All were retrospective studies, including 5 English articles and 5 Chinese articles, involving 300 patients. Literature screening procedure was presented in Figure 1.

Ten pieces of literature were included in this meta-analysis, and the basic characteristics of the study are shown in Table 1. The quality of the included studies was evaluated, with two articles assessed as grade A, five reports evaluated as grade B, and only three articles assessed as grade C, suggesting that the overall quality of the included articles was high.

#### 3.1.1. Meta-Analysis of Diagnostic Efficacy

Seven studies reported ^18^F-FDG PET/CT in the differential diagnosis of the benign and malignant hemophagocytic syndrome, with a pooled sensitivity of 0.82 (95% CI: 0.67–0.95), a specificity of 0.72 (95% CI: 0.51–0.86), a positive likelihood ratio of 2.89 (95% CI: 1.46–5.75), a positive likelihood ratio of 0.25 (95% CI: 0.12–0.54), and a diagnostic odds ratio of 2.89 (95% CI: 1.46–5.75), as shown in Figures 2, 3, and 4. The heterogeneity test results showed that *I*^2^ of sensitivity was 76.19%, *I*^2^ of specificity was 69.50%, *I*^2^ of positive likelihood ratio was 78.95%, *I*^2^ of negative likelihood ratio was 76.97%, and *I*^2^ of diagnostic odds ratio was 71.8%, suggesting high heterogeneity in sensitivity, specificity, positive likelihood ratio, negative likelihood ratio, and diagnostic odds ratio. The sensitivity analysis was performed for the included studies. After sensitivity analysis and outlier detection, no main source leading to increased heterogeneity was found. After excluding any literature, the effect on the results of the combined model was small, and the obtained results were relatively stable.

The article "Differential Diagnosis of Hemophagocytic Syndrome by 18F-FDG PET/CT: A Meta-Analysis" was retracted in 2023. Reasons: signs of a paper mill; suspected computer-generated content; unreliable results or conclusions; lack of ethics approval or compliance.

#### 3.1.2. SROC Curve Analysis

After SROC curve analysis of the data of the seven included articles, the results showed that the AUC was 0.84 (95% CI: 0.81–0.87), suggesting a high accuracy of ^18^F-FDG PET/CT in the differential diagnosis of benign and malignant hemophagocytic syndrome.  Figure 5.

#### 3.1.3. Publication Bias

Publication bias was detected for the included studies, and Deek's test results showed that *P*=0.97 (*P* > 0.05), suggesting that there was no publication bias in this meta-analysis.  Figure 6 is Deek's diagram. The *x*-axis was the diagnostic odds ratio, and the *y*-axis showed the 1/root.

#### 3.1.4. Meta-Analysis of SUVmax in Liver, Spleen, Lymph Nodes, and Bone Marrow of Patients with Benign and Malignant HPS

According to different organ and tissue sites, the differences of SUVmax values in the liver, spleen, lymph nodes, and bone marrow of patients with benign and malignant HPS were analyzed. In the analysis of the spleen, the SUVmax value in the spleen of patients with malignant HPS was significantly higher than that of patients with benign HPS, and the difference was statistically significant (MD = 3.43, 95% CI (2.47, 4.40), *P* < 0.05); in the analysis of bone marrow, the SUVmax value in the bone marrow of patients with malignant HPS was significantly higher than that of patients with benign HPS, and the difference was statistically significant (MD = 3.25, 95% CI (0.89, 5.61), *P* < 0.05); in the analysis of lymph nodes, the SUVmax value in the lymph nodes of patients with malignant HPS was significantly higher than that of patients with benign HPS, and the difference was statistically significant (MD = 3.68, 95% CI (1.45, 5.91), *P* < 0.05); in the analysis of liver, the SUVmax value in the liver of patients with malignant HPS was not significantly different from that of patients with benign HPS (MD = 0.10, 95% CI (−0.71, 0.91), *P* > 0.05).  Figure 7 is the forest map of SUVmax comparison in the liver, spleen, lymph nodes, and bone marrow of patients with benign and malignant HSP.

The article "Differential Diagnosis of Hemophagocytic Syndrome by 18F-FDG PET/CT: A Meta-Analysis" was retracted in 2023. Reasons: signs of a paper mill; suspected computer-generated content; unreliable results or conclusions; lack of ethics approval or compliance.

#### 3.1.5. Meta-Analysis of SUVmax in Liver, Spleen, Lymph Nodes, and Bone Marrow of Patients with HPS

According to the location of organs and tissues, the SUVmax values in the liver, spleen, lymph nodes, and bone marrow of HPS patients were analyzed. In the analysis of the spleen, the SUVmax in the spleen of HPS patients was 4.37 (95% CI: 3.97–4.78); in the study of bone marrow, the SUVmax in the spleen of HPS patients was 4.62 (95% CI: 4.21–5.04); in the analysis of lymph nodes, the SUVmax in the spleen of HPS patients was 6.55 (95% CI: 4.94–8.16); in the study of liver, the SUVmax in the spleen of HPS patients was 2.96 (95% CI: 1.19–4.73).  Figure 8 is the forest map of SUVmax comparison in the liver, spleen, lymph nodes, and bone marrow of HSP patients.

## 4. Discussion

HPS is a rare disease that usually occurs in infants and young children. It may also occur in adults. Children usually inherit the disease. In adults, many different conditions, including infections and cancer, can cause HPS. In this study, we found that ^18^F-FDG PET/CT was of great value in the diagnosis of HPS, and the SUVmax of HPS patients was more significant than 2.5, suggesting the presence of abnormalities; it had high accuracy, high sensitivity, and slightly poor specificity in the differential diagnosis of benign and malignant HPS and could effectively differentiate malignant HPS; meanwhile, it was found that the SUVmax values of the liver, spleen, lymph nodes, and bone marrow tissues after ^18^F-FDG PET/CT scan in patients with malignant HPS were significantly higher than those in patients with benign HPS, suggesting that malignant factors may cause the source of HPS in patients with SUVmax.

Currently, treatment options for HPS mainly rely on clinical experience and expert consensus. There is a lack of evidence from randomized controlled trials, treatment options are diverse, and close monitoring of treatment outcomes is required [27]. Studies have found that the treatment for HPS is mainly based on HLH-2004 treatment guidelines[28], and the combination of dexamethasone + etoposide + cyclosporine A is the initial treatment and maintenance treatment. The initial treatment is to inhibit T cell activation and macrophage function, thereby reducing the production of cytokine storm, which in turn alleviates the condition and reduces acute death. Some researchers [29] have reported that, with the use of liposomal adriamycin + etoposide + methylprednisolone in the treatment of 63 adult patients with relapsed HPS, the overall response rate was 76.2%, and complete remission was 27.0%, thus providing these patients with the opportunity to prolong survival and obtain further treatment of the primary disease or hematopoietic stem cell transplantation.

The article "Differential Diagnosis of Hemophagocytic Syndrome by 18F-FDG PET/CT: A Meta-Analysis" was retracted in 2023. Reasons: signs of a paper mill; suspected computer-generated content; unreliable results or conclusions; lack of ethics approval or compliance.

Furthermore, studies have confirmed that, for lymphoma patients with Epstein-Barr virus infection, the combination of CD20 monoclonal antibody therapy is recommended. At the same time, anti-CD52 antibodies and anti-IL-1 antibodies have also been reported for salvage therapy in HPS patients in recent years. Still, the remission rate is low, and only some patients can achieve partial remission [30].

According to the relevant HPS prognosis report, HPS treatment has poor prognosis response, high mortality, and short survival; especially, malignant tumor-related hemophagocytic syndrome has the worst prognosis. Data [31] showed that, through retrospective analysis of 40 patients with HPS, it was found that the mortality rate of patients in the malignant tumor group was significantly higher than that in the nonmalignant tumor group within a period. The presence of HPS in patients with malignant lymphoma is an important indicator of poor prognosis (body temperature, spleen size, blood cell count, ferritin, fibrinogen, and sCD25) [32]. Therefore, early and correct diagnosis plays a decisive role in the treatment and prognosis of the disease [33].

In recent years, with the rapid development of functional imaging techniques, 18F-FDG PET/CT, as whole-body metabolic imaging, can accurately show the extent involved by the lesion. A study has reported [34] that ^18^FPET/CT is helpful in the localization of bone marrow biopsy, especially in patients whose etiology still cannot be found by multiple aspirations. Studies have found that the most common manifestations of HPS on ^18^F-FDG PET/CT are hepatosplenic enlargement and increased FDG uptake, increased diffuse FDG uptake in the bone marrow, and higher FDG uptake in the spleen than in the liver [14, 35]. In HPS, increased FDG uptake in the spleen can more directly reflect immune cell activation, so the metabolism of the spleen can more precisely reflect the activity of systemic inflammation in HPS relative to the bone marrow. In addition, it has been shown that the mean SUV value ratio (SLRmean) of the spleen to the liver can be used to differentiate autoimmune diseases from uncomplicated localized infections [36]. A study [24] has found that FDG uptake in the liver of acute myelogenous leukemia (AML) is usually normal or slightly low.

In contrast, FDG uptake in the liver of AML-associated HPS is significantly higher. Therefore, the metabolic pattern of FDG on ^18^F-FDG PET/CT can be an important supplement to the clinical manifestations and laboratory parameters of HPS. Studies have confirmed that HPS associated with clinical and hematological malignancies has increased hepatomegaly, splenomegaly, and bone marrow uptake. Studies have shown that the SUVmax values of infection-related HPS are autoimmune disease-related HPS, and malignant tumor-related HPS is also significantly increased in turn [24, 37]. The FDG uptake in lymph nodes and spleen of malignant tumor-related HPS was significantly higher than that of nonmalignant tumor-related HPS. The cut-off value of SUVmax of lymph nodes was 3.3, and that of the spleen was about 3.4–4.8. ^18^F-FDG PET/CT showed hypermetabolism of the liver, spleen, and bone marrow, suggesting the possibility of lymphoma [37], and in addition, delayed ^18^F-FDG PET/CT imaging may help differentiate malignant lymphoma-associated HPS after a while: FDG uptake will be significantly increased in delayed imaging of malignant lymph nodes, while benign lymph nodes remain unchanged [38]. It has been reported that the diagnosis of HPS is based on a series of clinical, laboratory, immunological, and histopathological tests. Still, each test result lacks specificity, especially for diagnosing the primary disease and prognostic evaluation in patients with secondary HPS. This study is similar to most reports. Malignant lesions are more similar to nonmalignant lesions. Still, tumor-related groups are accompanied mainly by lymphadenopathy and often present with multiple and multiple lymph node enlargements throughout the body. The uptake degree of imaging agents is higher than nonmalignant lesions, which may be related to reactive lymph node hyperplasia in nonmalignant lesions. CT alone is not easy to distinguish, and biopsy of lymph nodes with significant imaging agent uptake on ^18^F-FDG PET/CT can guide more accurate and timely clinical etiological diagnosis. At the same time, the mean SUVmax in the malignant lesion group is significantly higher than that in the nonmalignant lesion group. Bone marrow and spleen infiltration of lymphoma can promote a higher degree of imaging agent uptake [39], which is helpful for differentiation to some extent. Additionally, there were several studies that showed that PET/CT is helpful for identifying the possible trigger (infection or malignant disease) and the extent of secondary HLH [40–43]. There were also some single-arm studies that showed that the ^18^F-FDG PET/CT especially played an important role in the differential diagnosis of HPS [44–46]. What is more, ^18^F-FDG PET/CT was useful for detecting underlying malignancy, and PET parameters correlated with laboratory parameters that reflected inflammatory status. ^18^F-FDG PET/CT might provide prognostic information for the management of patients with HPS.

The article "Differential Diagnosis of Hemophagocytic Syndrome by 18F-FDG PET/CT: A Meta-Analysis" was retracted in 2023. Reasons: signs of a paper mill; suspected computer-generated content; unreliable results or conclusions; lack of ethics approval or compliance.

In summary, HPS has complex etiology, diverse clinical manifestations, and rapid changes in the condition, is more critical, and has a high mortality rate, and its diagnosis and treatment are challenging. As a systemic and pathological examination, ^18^F-FDG PET/CT is of great significance in patients with HPS whose diagnosis is unknown, and there is no pathological confirmation. ^18^F-FDG PET/CT findings can reflect the location and activity of inflammatory lesions, thus supporting clinical diagnosis, helping to detect the potential cause of HPS, further guiding the biopsy site to identify the pathology, and assisting in determining the treatment plan; it is helpful to monitor the efficacy and has potential prognostic value.

In this study, we analyzed the diagnostic value of ^18^F-FDG PET/CT in the differential diagnosis of HPS, further confirming that ^18^F-FDG PET/CT is an effective means of diagnosing HPS and differentiating benign from malignant HPS. Thus, the conclusion obtained in this study is more persuasive than the results reported in single literature and can provide some guiding value for clinical diagnosis. However, this study also has some limitations. First, this study failed to find the cut-off value for the diagnosis of HPS and differential diagnosis of benign and malignant HPS, which makes ^18^F-FDG PET/CT still suffer from some limitations in the diagnosis of HPS; second, most of the studies included in this meta-analysis had relevant reports of SUV values but did not give specific SUV values but studied the correlation between SUV and some serum parameters, resulting in fewer literature data in this meta-analysis when analyzing SUV differences in the liver, spleen, lymph nodes, and bone marrow, affecting the reliability of the results. Third, the overall number of patients included in this study is also small, making the conclusions derived from a small sample size. Fourth, all of the included studies were retrospectively designed; this meta-analysis would have the limitations of the retrospective studies.

## 5. Conclusion

According to the data of existing literature, ^18^F-FDG PET/CT can be found to be an effective means of diagnosing HPS, while the differential diagnosis of the benign and malignant hemophagocytic syndrome also has high accuracy.

## Figures and Tables

**Figure 1:** Flowchart of literature search and screening.

**Figure 2:** Forest map of 18F-FDG PET/CT in the differential diagnosis of benign and malignant hemophagocytic syndrome.

The article "Differential Diagnosis of Hemophagocytic Syndrome by 18F-FDG PET/CT: A Meta-Analysis" was retracted in 2023. Reasons: signs of a paper mill; suspected computer-generated content; unreliable results or conclusions; lack of ethics approval or compliance.

**Figure 3:** Forest plot of likelihood ratio of ^18^F-FDG PET/CT in the differential diagnosis of benign and malignant hemophagocytic syndrome.

**Figure 4:** Forest map of the diagnostic odds ratio of ^18^F-FDG PET/CT in the differential diagnosis of benign and malignant hemophagocytic syndrome.

**Figure 5:** SROC curve of 18F-FDG PET/CT in the differential diagnosis of benign and malignant hemophagocytic syndrome.

**Figure 6:** Deek's diagram of 18F-FDG PET/CT in the differential diagnosis of benign and malignant hemophagocytic syndrome.

**Figure 7:** Forest map of SUVmax comparison in liver, spleen, lymph nodes, and bone marrow of patients with benign and malignant HSP.

**Figure 8:** Forest map of SUVmax comparison in liver, spleen, lymph nodes, and bone marrow of HSP patients.

**Table 1:** Basic characteristics and quality evaluation results of the included literature.

Study	Year	Country	Type of study	Gender (M/F)	Age	Sample sizes	PET/CT	Gold standard	Diagnostic criteria	Outcomes	Quality assessment
Qin xu et al.	2018	China	Retrospective study	21/14	15–65	35	18F-FDG	Pathological examination	HLH-2004	①②	B
Xin Liu et al.	2021	China	Retrospective study	19/18	17–79	37	18F-FDG	Pathological examination	HLH-2004	①	A
Xingbing Wang et al.	2014	China	Retrospective study	5/6	19–70	11	18F-FDG	Pathological examination	HLH-2004	①	B
Shuo Li et al.	2013	China	Retrospective study	18/12	14–70	30	18F-FDG	Pathological examination	HLH-2004	①	C
Liangyu Qi et al.	2019	China	Retrospective study	21/17	9–76	38	18F-FDG	Pathological examination	HLH-2004	①②	C
Yiu C R et al.	2011	China	Retrospective study	3/0	47–65	3	18F-FDG	Pathological examination	HLH-2004	②	C
Jahae Kim et al.	2013	Korea	Retrospective study	6/8	48–73	14	18F-FDG	Pathological examination	HLH-2004	①	B
Y. Zheng et al.	2016	China	Retrospective study	20/23	14–79	43	18F-FDG	Pathological examination	HLH-2004	①	B
Jujuan Wang et al.	2016	China	Retrospective study	NA	29–60	44	18F-FDG	Pathological examination	HLH-2004	②	A
Leilei Yuan et al.	2016	China	Retrospective study	28/17	17–79	45	18F-FDG	Pathological examination	HLH-2004	①	B

M: male; F: female; NA: not available; d: day; m: month; y: year; 1: maximum standardized uptake value (SUVmax); 2: diagnostic efficacy.

## Data Availability

The simulation experiment data used to support the findings of this study are available from the corresponding author upon request.
